The article "A Comparison of the Antiosteoporotic Effects of Cornelian Cherry (Cornus mas L.) Extracts from Red and Yellow Fruits Containing Different Constituents of Polyphenols and Iridoids in Osteoblasts and Osteoclasts" was published in 2022. Journal: Oxid Med Cell Longev.

# A Comparison of the Antiosteoporotic Effects of Cornelian Cherry (*Cornus mas* L.) Extracts from Red and Yellow Fruits Containing Different Constituents of Polyphenols and Iridoids in Osteoblasts and Osteoclasts

**DOI:** 10.1155/2022/4122253

**Published:** 2022-10-03

**Authors:** Eunkuk Park, Tomasz Sozański, Chang-Gun Lee, Alicja Z. Kucharska, Dominika Przybylska, Narcyz Piórecki, Seon-Yong Jeong

**Affiliations:** ^1^Department of Medical Genetics, Ajou University School of Medicine, Suwon 16499, Republic of Korea; ^2^Department of Pharmacology, Wroclaw Medical University, ul. J. Mikulicza-Radeckiego 2, 50-345 Wroclaw, Poland; ^3^AI-Superconvergence KIURI Translational Research Center, Ajou University School of Medicine, Suwon 16499, Republic of Korea; ^4^Department of Fruit, Vegetable and Plant Nutraceutical Technology, Wroclaw University of Environmental and Life Sciences, J. Chełmońskiego 37, 51-630 Wroclaw, Poland; ^5^Bolestraszyce Arboretum and Institute of Physiography, Bolestraszyce 130, 37-722 Wyszatyce, Poland; ^6^Institute of Physical Culture Sciences, Medical College, University of Rzeszów, Cicha 2A, 35-326 Rzeszów, Poland

## Abstract

**Methods:**

Polyphenolic and iridoid constituents of extracts were analyzed qualitatively and quantitatively using the ultraperformance liquid chromatography system coupled with a quadrupole-time of flight mass spectrometry. Primary cultured osteoblasts isolated from mouse calvarias and osteoclast-lineage primary cultured monocytes isolated from mouse bone marrow were used for the assessment of osteoblast and osteoclast differentiation. In the osteoblast culture, cellular viability, alkaline phosphatase (ALP) activity, ALP staining, and mRNA expression of Alpl and Runx2 were examined. In the osteoclast culture, the examined parameters were cellular viability, tartrate-resistant acid phosphatase (TRAP) activity and staining, and mRNA expression of Nfatc1, Ctsk, and Acp.

**Results:**

A total of 41 main compounds of iridoids, anthocyanins, hydrolysable tannins, phenolic acids, and flavonols were identified in the three extracts. RED EXT1 contained most of the tested polyphenols and iridoids and was the only extract containing anthocyanins. YL EXT2 contained only one iridoid, loganic acid and gallic acid. YL EXT3 comprised a mixture of iridoids and polyphenols. RED EXT1, YL EXT 2, and to a lesser extent YL EXT3 promoted osteoblast differentiation increasing significantly ALP activity and the amount of ALP-positive stained cells. All extracts upregulated mRNA expression of Alpl and Runx2. RED EXT1 caused the most significant decrease in TRAP activity and the numbers of TRAP-positive multinucleated cells. RED EXT1 caused also the most significant downregulation of mRNA expression of osteoclast related genes Nfatc1, Ctsk, and Acp5. Extracts from yellow fruits, mostly YL EXT2 caused lower, but still significant inhibitory effect on TRAP and osteoclast related genes.

The article "A Comparison of the Antiosteoporotic Effects of Cornelian Cherry (Cornus mas L.) Extracts from Red and Yellow Fruits Containing Different Constituents of Polyphenols and Iridoids in Osteoblasts and Osteoclasts" was published in 2022. Journal: Oxid Med Cell Longev.

**Conclusions:**

The main conclusion of our study is that all three extracts, especially RED EXT1 from red cornelian cherry fruits, possess the antiosteoporotic potential and may be a promising phytomedicine candidate for the prevention and treatment of osteoporosis.

## 1. Introduction

Osteoporosis is a common systemic bone disease characterized by the loss of bone mass and deterioration of the bone microstructure, leading to fractures and subsequent complications. An increased life expectancy in developed countries combined with comorbidities and drugs causing bone loss has resulted in osteoporosis, becoming more prominent in the last few decades. Moreover, increased levels of physical activity in elderly populations, offering several benefits but leading to a higher risk of pathological fractures, makes osteoporosis an increasingly greater medical, social, and economic challenge.

Bone remodeling is regulated by homeostasis between osteoclasts resorbing old or damaged bone cells and osteoblasts developing new bone structures [1]. The differentiation and function of osteoclasts and osteoblasts are key target areas for antiosteoporotic agents. It has been proven that bone metabolism can be modulated by nutrients [2, 3]. Recently published studies have reported that polyphenols, especially anthocyanins [4, 5], phenolic acids [6], and flavonols [7], as well as iridoids [8] and hydrolysable tannins [9] can prevent bone loss through different mechanisms. All these substances are present in cornelian cherries, in varying amounts, making their extracts promising candidates for antiosteoporotic agents.

A previous *in vitro* study demonstrated that *Cornus officinalis* Sieb. et Zucc. shared a few similar iridoid and polyphenol constituents with the cornelian cherry (*Cornus mas* L.), and it inhibits the receptor activator of nuclear factor-kappaB ligand (RANKL)-induced osteoclast differentiation [10]. Our previous studies showed that red cornelian cherries, rich in polyphenols and iridoids, prevented both cholesterol-induced dyslipidemia and atherosclerosis via the upregulation of peroxisome proliferator-activated receptors (PPARs) expression [11–14] and prevented bone loss in osteoporotic animals by inhibiting bone resorption and increasing bone formation [15]. Another study demonstrated that the pulp of cornelian cherries partially reversed impaired microarchitecture bone quality in Zucker diabetic fatty rats [16].

The article "A Comparison of the Antiosteoporotic Effects of Cornelian Cherry (Cornus mas L.) Extracts from Red and Yellow Fruits Containing Different Constituents of Polyphenols and Iridoids in Osteoblasts and Osteoclasts" was published in 2022. Journal: Oxid Med Cell Longev.

In the present study, we have compared the antiosteoporotic effects of three different extracts from cornelian cherry fruits: RED EXT1 from red fruits containing exceptionally anthocyanins and substantial amounts of various other polyphenols and iridoids, YL EXT2 from yellow fruits containing a single iridoid, loganic acid and gallic acid, and YL EXT3 from yellow fruits comprising substantial amounts of various iridoids and polyphenols. To investigate the effects of extracts on bone remodeling, we used an *in vitro* model of mouse primary cultured osteoblasts isolated from mouse calvarias and osteoclasts isolated from mouse bone marrow monocytes. In the osteoblast culture, the analyzed parameters were cellular viability, alkaline phosphatase (ALP) activity and amount of ALP-positive stained cells, and mRNA expression of a gene (Alpl) and transcription factor (Runx2) involved in osteoblastic bone remodeling. In osteoclast culture, the analysis pertained to cellular viability, tartrate-resistant acid phosphatase (TRAP) activity, the number of TRAP-positive multinucleated cells, and mRNA expression of transcriptional factor (Ctsk), as well as genes (Nfatc1, Acp5) involved in osteoclast differentiation and activity.

## 2. Materials and Methods

### 2.1. Reagents and Standards

All reagents and organic solvents were of analytical grade. Authentic standards of loganic acid, loganin, sweroside, cyanidin 3-*O*-glucoside, *p*-coumaric acid, ellagic acid, quercetin 3-*O*-glucoside, and kaempferol 3-*O*-glucoside were purchased from Extrasynthese (Genay, France). *Trans*-caftaric acid was purchased from the Cayman Chemical Company (Michigan, EUA, Ann Arbor, MI, USA). *Trans*-coutaric acid was purchased from Merck (Darmstadt, Germany). Methanol, acetonitrile, and formic acid were obtained from POCH (Gliwice, Poland).

### 2.2. Extraction, Purification, and Fractionation of Extracts

Red (‘Podolski') and yellow (‘Yantarnyi' and ‘Flava') cornelian cherries were harvested in the Arboretum in Bolestraszyce, near Przemyśl, Poland. The plant materials were authenticated by Elżbieta Żygała, M.Sc. (Arboretum and Institute of Physiography in Bolestraszyce, Przemyśl, Poland), and adequate voucher specimens (‘Yantarnyi' – BDPA 14131; ‘Flava' – BDPA 8795; ‘Podolski' – BDPA 10462) were deposited at the Herbariums of Arboretum in Bolestraszyce, Poland. After harvesting, the fruits were immediately frozen at −20°C.

Extracts were prepared as previously described by Lewandowski et al. [17] with some modifications. Frozen ripe cornelian cherries were shredded and heated for 5 min at 95°C using a Thermomix (Vorwerk, Wuppertal, Germany). The pulp was subsequently cooled to 50°C and depectinized at this temperature for 2 h by adding 0.5 mL/kg of Pectinex BE XXL (Novozymes A/S, Denmark). After depectinization, the pulp was pressed in a laboratory hydraulic press (SRSE, Warsaw, Poland). The pressed juice was filtered and run through an Amberlite XAD-16 resin column (Rohm and Haas, Chauny Cedex, France). Impurities were washed off with distilled water. RED EXT1 (red fruits) and YL EXT3 (yellow fruits) were eluted with 80% ethanol while YL EXT2 (yellow fruits) was eluted with up to 50% ethanol (v/v in water). The eluents were concentrated at 40°C under vacuum. The solvent was evaporated using a Rotavapor (Unipan, Warsaw, Poland) and freeze-dried (Alpha 1–4 LSC, Christ, Osterode am Harz, Germany). As a result, we have obtained three extracts from cornelian cherry fruits: RED EXT1 from red fruits containing substantial amounts of various anthocyanins, iridoids, and hydrolysable tannins with moderate or small amounts of phenolic acids and flavonols, YL EXT2 from yellow fruits containing a single iridoid, loganic acid and small amounts of phenolic acids, and YL EXT3 from yellow fruits comprising substantial amounts of various iridoids and hydrolysable tannins, and moderate or small amounts of phenolic acids and flavonols.

The article "A Comparison of the Antiosteoporotic Effects of Cornelian Cherry (Cornus mas L.) Extracts from Red and Yellow Fruits Containing Different Constituents of Polyphenols and Iridoids in Osteoblasts and Osteoclasts" was published in 2022. Journal: Oxid Med Cell Longev.

### 2.3. Qualitative Identification of Compounds by Liquid Chromatography-Mass Spectrometry (LC-MS)

This method was previously described by Przybylska et al. [18]. Compounds were identified using the Acquity ultraperformance liquid chromatography (UPLC) system, coupled with a quadrupole-time of flight (Q-TOF) MS instrument (UPLC/Synapt Q-TOF MS, Waters Corp., Milford, MA, USA), with an electrospray ionization source. Separation was achieved using an Acquity UPLC BEH C18 column (100 × 2.1 mm i.d., 1.7 *μ*m; Waters Corp., Milford, MA, USA). The mobile phase was a mixture of 2.0% aq. formic acid v/v (a) and acetonitrile (b). The gradient program is as follows: initial conditions: 1% B in A, 12 min; 25% B in A, 12.5 min; 100% B, 13.5 min; 1% B in A. The flow rate was 0.45 mL/min, and the injection volume was 5 *μ*L. The column was operated at 30°C. The UV-Vis absorption spectra were recorded online during the UPLC analysis, and the spectra were measured in the wavelength range of 200–600 nm, in steps of 2 nm. The major operating parameters of the Q-TOF MS were set as follows: capillary voltage of 2.0 kV, cone voltage of 40 V, cone gas flow of 11 L/h, collision energy of 28–30 eV, source temperature of 100°C, desolvation temperature of 250°C, argon as the collision gas, desolvation gas (nitrogen) flow rate of 600 L/h, and data acquisition range (*m/z*) of 100–2500 Da. The compounds were monitored at 245, 280, 320, 360, and 520 nm and explored in the negative and positive (only anthocyanins) modes before and after fragmentation. The data was collected with the MassLynx V 4.1 software (Waters Corp., Milford, MA, USA).

The article "A Comparison of the Antiosteoporotic Effects of Cornelian Cherry (Cornus mas L.) Extracts from Red and Yellow Fruits Containing Different Constituents of Polyphenols and Iridoids in Osteoblasts and Osteoclasts" was published in 2022. Journal: Oxid Med Cell Longev.

### 2.4. Quantitative Determination of Anthocyanins, Flavonols, Phenolic Acids, and Iridoids Using HPLC-PDA

The HPLC analysis was performed as described by Spychaj et al. [19] using the Dionex (Germering, Germany) system equipped with an Ultimate 3000 diode array detector, LPG-3400A quaternary pump, EWPS-3000SI autosampler, TCC-3000SD thermostated column compartment, and controlled with the Chromeleon v.7.2 software. Separation was achieved using a Cadenza Imtakt column CD-C18 (75 × 4.6 mm, 5 *μ*m). The mobile phase was composed of solvent A (4.5% aq. formic acid, v/v) and solvent B (100% acetonitrile). The gradient profile is as follows: 5% B in A, 0–1 min; 25% B in A, 1–20 min; 100% B, 20–26 min; 5% B in A, 26–30 min. The flow rate of the mobile phase was 1 mL/min, and the injection volume was 20 *μ*L. The column was operated at 30°C. Anthocyanins were detected at 520 nm, flavonols at 360 nm, phenolic acids at 320 nm, gallic acid at 280 nm, ellagic acid at 254 nm, and iridoids at 245 nm. Calibration curves at concentrations ranging from 0.02 to 0.3 mg/mL (*R*^2^ ≥ 0.9998) were determined experimentally for cyanidin 3-*O*-glucoside, quercetin 3-*O*-glucoside, kaempferol 3-glucoside, caffeic acid, *trans*-caftaric acid, trans-coutaric acid, *p*-coumaric acid, ellagic acid, and gallic acid. The results were expressed as mg/100 g of the dried extract. Results were provided as the mean ± standard deviation of three replications and expressed as mg/100 g dw (dry weight) of the extract.

### 2.5. Quantitative Determination of Hydrolysable Tannins by HPLC-PDA

The HPLC analysis was performed as described by Przybylska et al. [18] using the Dionex (Germering, Germany) system equipped with an Ultimate 3000 diode array detector, LPG-3400A quaternary pump, EWPS-3000SI autosampler, TCC-3000SD thermostated column compartment, and controlled using the Chromeleon v.7.2 software. Separation was achieved using a Hypersil GOLD C18-column (250 × 4.6 mm, 5 *μ*m; Thermo Fisher Scientific Inc., UK). The following mixtures were used as eluents: (a), water-FA (98.5 : 1.5, v/v) and (b), acetonitrile-FA (98.5 : 1.5, v/v). The gradient profile is as follows: initial conditions: 100% A, 30 min; 30% B, 33 min; 70% B, 45 min; 70% B in A, 48 min; 100% B, 55–60 min; 100% A. The flow rate of the mobile phase was 1.2 mL/min, and the injection volume was 20 *μ*L. The column was operated at 22°C. Hydrolysable tannins were detected at 280 nm. A calibration curve at concentrations ranging from 0.02 to 0.3 mg/mL (*R*^2^ ≥ 0.9996) was determined experimentally for gallic acid. Results are provided as the total of individual isomers of three replications and expressed as mg/100 g of the extract.

The article "A Comparison of the Antiosteoporotic Effects of Cornelian Cherry (Cornus mas L.) Extracts from Red and Yellow Fruits Containing Different Constituents of Polyphenols and Iridoids in Osteoblasts and Osteoclasts" was published in 2022. Journal: Oxid Med Cell Longev.

### 2.6. Primary Osteoblast Culture and Induction of Osteoblast Differentiation

Primary cell cultures of the mice were conducted using a protocol approved by the Institutional Animal Care and Use Committee (IACUC) of Ajou University School of Medicine (2016-0062). Primary osteoblasts of the mice were isolated from neonatal C57BL/6 mice (4–5 pups), as previously described [20]. The calvarias of the mice were dissected and digested with collagenase II (Sigma, St. Louis, MO, USA) at 37°C for 2 h. The digestive solution was filtered through a 40 *μ*m cell strainer, and the cells were incubated with an *α*-modified minimal essential medium (*α*-MEM; Gibco) supplemented with 10% fetal bovine serum (FBS; Gibco) and 1% penicillin/streptomycin (Gibco) for 2–3 days. After 70–80% of confluency was reached, the cells were incubated with 10 mM *β*-glycerophosphate (Sigma) and 50 *μ*g/mL ascorbic acid (Sigma) for 3 days.

### 2.7. Isolation of Primary Monocytes and Induction of Osteoclast Differentiation

To isolate osteoclast-lineage primary-cultured monocytes, bone marrow (BM) cells from nine-week-old C57BL/6 mice were isolated as previously described [21]. The femoral bones of the mice were flushed using warm phosphate-buffered saline (Gibco), and the cellular suspension was subsequently filtered through a 40 *μ*m cell strainer to remove the debris. BM cells were then incubated with an *α*-MEM (Gibco) containing 10% FBS (Gibco) and 50 ng/mL of macrophage colony-stimulating factor (M-CSF) (Peprotech, Cranbury, NJ, USA) without penicillin/streptomycin (Gibco) for 3 days in a petri dish. For osteoclast differentiation, the cells were seeded in a 96-well plate and incubated with a growth medium supplemented with M-CSF (50 ng/mL; Peprotech) and RANKL (50 ng/mL; Peprotech) for 5 days.

### 2.8. Cell Viability Assay

The cells were incubated in 96-well plates and treated with different concentrations of *Cornus mas* L. extracts (2, 5, and 10 *μ*g/mL) during differentiation. The cells were then incubated with D-Plus™ cell counting kit (CCK) cell viability assay reagent (Dongin Biotech, Seoul, Korea) at 37°C, and the cell viability was measured using a microplate reader (Bio-Rad, Hercules, CA, USA) at an absorbance of 450 nm.

### 2.9. ALP/TRAP Activity Assay and Staining

The cells were collected using a lysis buffer (0.5 M Tris-hydrogen chloride (HCL), pH 8.8, containing 0.9% sodium chloride, 1% Triton X-100, and 200 mM ethylenediaminetetraacetic acid (EDTA)), and ALP activity was measured using 1-Step™ p-nitrophenyl phosphate (Sigma) according to the manufacturer's recommendations. ALP-positive cells were stained with 5-bromo-4-chloro-3-indolyl phosphate/nitro blue tetrazolium (BCIP/NBT; Sigma) at room temperature. TRAP activity and staining were processed using an Acid Phosphatase Kit (Sigma) in accordance with the manufacturer's instructions.

The article "A Comparison of the Antiosteoporotic Effects of Cornelian Cherry (Cornus mas L.) Extracts from Red and Yellow Fruits Containing Different Constituents of Polyphenols and Iridoids in Osteoblasts and Osteoclasts" was published in 2022. Journal: Oxid Med Cell Longev.

### 2.10. Quantitative Reverse-Transcriptase Polymerase Chain Reaction (qRT-PCR)

The total RNA was isolated using the TRIzol reagent (Invitrogen, Carlsbad, CA, USA) according to the manufacturer's instruction, and the complementary DNA (cDNA) was synthesized using a RevertAid™ H Minus First Strand cDNA Synthesis Kit (Fermentas, Hanover, NH, USA). qRT-PCR was processed using a SYBR Green I qPCR Kit (TaKaRa, Shiga, Japan), via the CFX Connect™ Real-Time System (Bio-Rad). The gene-specific primers used in this study were as follows: forward 5′-TCC CAC GTT TTC ACA TTC GG-3′ and reverse 5′-CCC GTT ACC ATA TAG GAT AGC C-3′ for mouse Alpl, forward 5′-TAA AGT GAC AGT GGA CGG TCC C-3′ and reverse 5′-AAT GCG CCC TAA ATC ACT GAG G-3′ for mouse Runx2, forward 5′-AAT ACC TCC CTC TCG ATC CTA CA-3′ and reverse 5′-TGG TTC TTG ACT GGA GTA ACG TA-3′ for mouse Ctsk, forward 5′-TGG TAT GTG CTG GCT GGA AAC-3′ and reverse 5′-AGT TGC CAC ACA GCA TCA CTG-3′ for mouse Acp5, forward 5′-AGG TCG GTG TGA ACG GAT TTG-3′ and reverse 5′-TGT AGA CCA TGT AGT TGA GGT CA-3′ for mouse Gapdh, forward 5′-GAG GAG TCC TGT TGA TGT TGC CAG-3′ and reverse 5′-GGC TGG CCT ATA GGC TCA TAG TGC-3′ for mouse Hprt. All gene expression levels were normalized using mouse Gapdh (osteoblast) and mouse Hprt (osteoclast), and relative expression levels were calculated using the 2^−ΔΔCt^ method (ΔΔCt = ΔCt_Treatment_ − ΔCt − _Induction_).

### 2.11. Statistical Analysis

The data in the bar graphs is presented as the mean ± standard error of the mean (SEM) using the GraphPad Prism 9.0 software (GraphPad Software, San Diego, CA, USA). Statistical analysis was performed in multiple groups using a one-way analysis of variance with Tukey's honest significant difference post hoc test. A probability value below 0.05 (*p* < 0.05) was considered statistically significant.

## 3. Results and Discussion

### 3.1. A Comparison of the Chemical Composition of Cornelian Cherry (*Cornus mas* L.) Extracts from Red and Yellow Fruits

The polyphenols and iridoids were analyzed via LC-MS and HPLC in the three extracts. The results of qualitative and quantitative identification of the compounds of cornelian cherry extracts are presented in Table 1.

Phenolic and iridoid compounds, as well as hydrolysable tannins, were identified by their elution order, retention times, spectra of individual peaks (MS, MS/MS), and by comparison with data in the literature [22–24]. A total of 41 main compounds were identified: 4 iridoids (loganic acid and cornuside with pseudomolecular ions [M − H]^−^ at *m/z* 375 and 541, respectively, and sweroside and loganin with [M − H + 46]^−^ at *m/z* 403 and 435, respectively), 7 anthocyanins (5 glycosides: delphinidin 3-*O*-galactoside, cyanidin 3-*O*-galactoside, cyanidin 3-*O*-robinobioside, pelargonidin 3-*O*-galactoside, and pelargonidin 3-*O*-robinobioside with [M + H]^+^ at *m/z* 463, 449, 595, 433, and 579, respectively, and 2 aglycons: cyanidin and pelargonidin with [M + H]^+^ at *m/z* 287 and 271, respectively), 6 phenolic acids (gallic acid, 2 isomers of caftaric acid, coutaric acid, *p*-coumaric acid, and ellagic acid with [M − H]^−^ at *m/z* 169, 311, 295, 163, and 301, respectively), 4 flavonols (quercetin 3-*O*-glucuronide, quercetin 3-*O*-glucoside, kaempferol 3-*O*-galactoside, and kaempferol 3-*O*-glucuronide with [M − H]^−^ at *m/z* 477, 463, 447, and 461, respectively), and 20 hydrolysable tannins, including their spatial isomers. Among the hydrolysable tannins, the main compounds were one trimeric ellagitannin (cornusiin C, which gave two ions, [M − 2H]^–2^ at *m/z* 1176 and [M − H]^–^ at *m/z* 2353), two dimeric ellagitannins (camptothin A, which displayed two ions [M − 2H]^–2^ at *m/z* 708 and [M − H]^–^ at *m/z* 1417 and cornusiin A with two ions, [M − 2H]^–2^ at *m/z* 784 and [M − H]^–^ at *m/z* 1569), as well as gemin D – the simplest among the ellagitannin molecules with ion [M − H]^−^ at *m*/*z* = 633 and its two derivatives (tellimagrandin I with [M − H]^−^ at *m/z* 785 and tellimagrandin II with [M − H]^−^ at *m/z* 937).

The article "A Comparison of the Antiosteoporotic Effects of Cornelian Cherry (Cornus mas L.) Extracts from Red and Yellow Fruits Containing Different Constituents of Polyphenols and Iridoids in Osteoblasts and Osteoclasts" was published in 2022. Journal: Oxid Med Cell Longev.

RED EXT1 contained most of the identified compounds (40 compounds), namely 16.9% iridoids, 3.5% anthocyanins, 1.2% phenolic acids, 0.6% flavonols, and 16.8% hydrolysable tannins. The quantitative and qualitative composition of iridoids and phenolic compounds in RED EXT1 is comparable to the composition of the red fruit extract described by Dzydzan et al. [23]. Extracts from yellow fruits (YL EXT2 and YL EXT3) did not contain anthocyanins but were richer in iridoids. YL EXT2 contained only one iridoid, 22.1% of loganic acid, whereas YL EXT3 contained four iridoids, which made up a quantity of 27.7% in total and included 17% of loganic acid. YL EXT2 contained four phenolic acids which made up a quantity of only 0.9% in total. As compared to the other extracts, YL EXT3 was the richest in phenolic acids, making up a quantity of 3.5% in total. The flavonols found in YL EXT3 were comparable to those present in RED EXT1, whereas YL EXT2 did not contain any of these compounds. A comparison between the two yellow fruit extracts showed that YL EXT2 mainly contained loganic acid and small amounts of phenolic acids, but no flavonols or tannins, whereas YL EXT3 was more abundant in various iridoids, phenolic acids, and hydrolysable tannins. Collectively, the three extracts contained different constituents of iridoids, anthocyanins, hydrolysable tannins, phenolic acids, and flavonols.

The article "A Comparison of the Antiosteoporotic Effects of Cornelian Cherry (Cornus mas L.) Extracts from Red and Yellow Fruits Containing Different Constituents of Polyphenols and Iridoids in Osteoblasts and Osteoclasts" was published in 2022. Journal: Oxid Med Cell Longev.

### 3.2. The Effects of Extracts from Cornelian Cherry Fruits on Osteoblast Differentiation

Further, we investigated the effects of the three cornelian cherries (*Cornus mas* L.) extracts (RED EXT1, YL EXT2, and YL EXT3) on osteoblast differentiation. Primary osteoblasts isolated from neonatal mouse calvarias were cultured in an osteoblastic induction media containing *β*-glycerophosphate and ascorbic acid and cotreated with different concentrations of *Cornus mas* L. extracts (2, 5, and 10 *μ*g/mL) for three days. Treatment with the extracts did not influence the cell viability of primary-cultured osteoblasts, proving that there is no risk of cytotoxicity from these three extracts for primary osteoblasts (Figure 1).

Osteoblast differentiation was evaluated using an ALP activity assay and ALP staining. ALP plays a major role in the regulation of bone formation and mineralization during osteoblast differentiation [25]. Treatment with two of the three extracts, RED EXT1 and YL EXT2, significantly increased ALP activity at a concentration of 5 and 10 *μ*g/mL. EXT3 increased ALP activity only at a concentration of 10 *μ*g/mL (Figure 2). In addition, ALP staining results also showed an increase in ALP staining-positive cells in all three extracts (Figure 3). Although all three cornelian cherry extracts augmented osteoblast differentiation by increasing ALP activity, RED EXT1 and YL EXT2, compared to the YL EXT3, exhibited better efficacy on both ALP activity and staining, probably due to differences in the contents of the bioactive compounds. RED EXT1 consisted of abundant amounts of anthocyanins, a mixture of iridoids and hydrolyzable tannins, moderate amounts of phenolic acids, and small amounts of flavonols. Notably, despite YL EXT2 containing only a single iridoid, loganic acid, and a few phenolic acids, it showed better efficacy than YL EXT3 containing various iridoids and polyphenols. Among the three extracts, only YL EXT2 consisted of gallic acid and the highest amount of loganic acid, suggesting that these two compounds may be responsible for the better effect of YL EXT2 on the augmentation of osteoblast differentiation.

Next, we further investigated the effect of the three extracts on the mRNA expression changes of osteoblastogenesis biomarker genes: Alpl and runt-related transcription factor 2 (Runx2). Alpl is a bone-specific isoform localized on the surface of osteoblasts and is a sensitive indicator of bone metabolism [26]. Runx2 is an essential transcription factor for osteoblast differentiation during the early stages of bone formation [27]. These factors play an important role in the transcriptional regulation of bone formation and mineralization [28]. Primary cultured preosteoblasts were treated with the three extracts (RED EXT1, YL EXT2, and YL EXT3) at 10 *μ*g/mL for 3 days, and thereafter the mRNA expression levels were analyzed using quantitative reverse transcriptase-polymerase chain reaction (qRT-PCR). All three extracts increased the mRNA expression levels of Alpl and Runx2 compared to that in the osteoblast-induced controls (Figure 4). These results suggest that *Cornus mas* L. extracts may enhance osteoblast differentiation by upregulating the expression of the Alpl and Runx2 genes at the transcription level. There was no difference in the augmentation efficacy of the three extracts for the expression of Alpl and Runx2. Taken together, these results showed that the three extracts from the *Cornus mas* L. fruits exhibited bone formation effects.

The article "A Comparison of the Antiosteoporotic Effects of Cornelian Cherry (Cornus mas L.) Extracts from Red and Yellow Fruits Containing Different Constituents of Polyphenols and Iridoids in Osteoblasts and Osteoclasts" was published in 2022. Journal: Oxid Med Cell Longev.

### 3.3. The Effects of Cornelian Cherry Fruits Extracts on Osteoclast Differentiation

Imbalanced homeostasis between bone resorption and bone formation results in weak and fragile bones associated with the risk of developing bone diseases [1, 29]. Dysregulation of osteoclast differentiation is a key factor causing abnormal bone metabolism and leading to osteoporosis [30–33]. Previous studies have suggested that a decrease in osteoclast differentiation is one of the main strategies for the prevention and treatment of osteoporosis [34–37]. Therefore, we investigated the effects of the three *Cornus mas* L. extracts (RED EXT1, YL EXT2, and YL EXT3) on osteoclast differentiation. Mouse bone marrow-derived osteoclast-lineage primary-cultured monocytes were isolated from the femoral bone. To induce osteoclast differentiation, the monocytes were treated with M-CSF and RANKL [38]. Treatment with the three extracts at three different concentrations (2, 5, and 10 *μ*g/mL) for 5 days did not affect cell viability, indicating that there is no risk of cytotoxicity for primary monocytes from these three extracts (Figure 5).

During osteoclast differentiation, TRAP stimulates the migration of osteoclasts into the bone resorption region [39]. TRAP is considered to be an important osteoclast histochemical indicator during skeletal development [40]. To assess osteoclast differentiation, TRAP activity assays and TRAP staining were used in this study. All three *Cornus mas* L. extracts showed a significant decrease in TRAP activity in the primary monocytes of mice at 10 *μ*g/mL, and RED EXT1 and YL EXT2 also showed a significant decrease at 2 and 5 *μ*g/mL (Figure 6). Among the three extracts, RED EXT1 exhibited the best efficacy, higher as compared to extracts from yellow fruits (Figure 6(a)). The results of the TRAP staining further revealed that the number of TRAP-positive multinuclear cells was significantly decreased after treatment with the three extracts (Figure 7). These results indicate that the *Cornus mas* L. extracts prevented osteoclast differentiation by decreasing TRAP activity, resulting in the attenuation of osteoclastic bone resorption. The best inhibitions of TRAP activity and TRAP staining were observed from the RED EXT1. Anthocyanins were only detected in RED EXT1, suggesting that the pronounce inhibitory effect of RED EXT1 on TRAP activity and staining could be attributed to the anthocyanins.

The article "A Comparison of the Antiosteoporotic Effects of Cornelian Cherry (Cornus mas L.) Extracts from Red and Yellow Fruits Containing Different Constituents of Polyphenols and Iridoids in Osteoblasts and Osteoclasts" was published in 2022. Journal: Oxid Med Cell Longev.

Bone resorption resulting from osteoclast differentiation is regulated by osteoclast-related enzymes, such as tartrate-resistant acid phosphatase 5 (Acp5) and cathepsin K (Ctsk) [41]. The transcription factor, nuclear factor of activated T cells 1 (Nfatc1), is known to promote osteoclast differentiation [42]. To confirm the inhibitory effects of *Cornus mas* L. extracts on osteoclast differentiation, the mRNA expression changes of osteoclastogenesis-related genes (Nfatc1, Ctsk, and Acp5) were investigated. The results showed that treatment with all three extracts significantly decreased the mRNA expression levels of Nfatc1, Ctsk, and Acp5 at a concentration of 10 *μ*g/mL (Figure 8). This finding indicates that *Cornus mas* L. extracts inhibit osteoclast differentiation through the decreased expression of these osteoclastogenic genes. Being consistent with the results from TRAP activity assays and staining, RED EXT1 was more effective than YL EXT2 and YL EXT3 in this experiment. These results suggest that the anthocyanins contained in RED EXT1 play a crucial role in the osteoclastogenesis reduction effects of *Cornus mas* L. extracts.

We analyzed and compared the constituents in a total of 41 compounds of iridoids, phenolic acids, flavonols, anthocyanins, and tannins in the three extracts obtained from red (RED EXT1) and yellow (YL EXT2 and YL EXT3) *Cornus mas* L. fruits using LC-MS and HPLC (Table 1). Although we did not examine the identified compounds directly, comparing the antiosteoporotic efficacies of the three extracts and reviewing the literature, it is possible to interpret which compounds are responsible for the antiosteoporotic effects of the extracts.

The article "A Comparison of the Antiosteoporotic Effects of Cornelian Cherry (Cornus mas L.) Extracts from Red and Yellow Fruits Containing Different Constituents of Polyphenols and Iridoids in Osteoblasts and Osteoclasts" was published in 2022. Journal: Oxid Med Cell Longev.

Our results are consistent with our recently published studies showing the antiosteoporotic effects of the cornelian cherry extract containing loganic acid. Park et al. [8] found that loganic acid isolated from *Gentiana lutea* L. roots extract significantly stimulated osteoblast differentiation by increasing ALP activity and upregulating the mRNA expression of Alpl, Bglap, and Sp7. In animal experiments, extracts from the cornelian cherry ameliorated the harmful changes in the bone turnover markers and bone mineral density (BMD) of hypercholesterolemic-diet rabbits [15] and counteracted the decrease in BMD and bone flexural strength of ovariectomized mice [8, 43]. In addition, phenolic acids, such as gallic acid and ellagic acid, were also revealed to have antiosteoporotic effects through the RANKL-related pathway [6, 44]. Unexpectedly, the antiosteoporotic effects of the YL EXT2 extract, containing only a single iridoid, loganic acid, were better than that of the YL EXT3 extract containing various iridoids including loganic acid, loganin, cornuside, and sweroside. Loganin and sweroside are known to have beneficial bone remodeling roles from previous studies [45, 46], and cornuside also reportedly has an antiosteoporotic effect [47]. We may try to explain the better antiosteoporotic effect of YL EXT2 because it contains uniquely gallic acid and a higher amount of loganic acid than YL EXT3. The exact molecular mechanism of the antiosteoporotic effect proposed for loganic acid requires further investigation, although anti-inflammatory activity and impact on described transcription factors and genes seem to be involved.

Regarding anthocyanins, although previous studies proved their possible inhibitory effect on osteoclast differentiation through the RANKL-mediated pathway [48, 49], only a few recently published studies suggest their possible enhanced effect on osteoblast differentiation and osteoblast-related mineralization through the ERK1/2 signaling pathway [50] or the inhibition of GSK-3*β* and subsequent activation of *β*-catenin [4]. Other proposed antiosteoporotic mechanisms of action of anthocyanins include their anti-inflammatory and antioxidant properties [50]. Inflammatory factors, glutathione depletion, and redox stress can inhibit the synthesis and differentiation of osteoblasts and bone mineralization. Polyphenols, especially anthocyanins can reduce these processes by the activation of sirtuin type 1 deacetylase expression with subsequent upregulation of ALP and Runx2 [51].

Phenolic acids, such as gallic acid or ellagic acid showed in other studies an antiosteoporotic effect through the RANKL-related pathway [6, 44]. Nevertheless, in our study, gallic acid was found only in small amounts in YL EXT2 and ellagic acid was present in small amounts in RED EXT1, and moderate amounts of it were found in YL EXT3. Cornelian cherry extracts, especially YL EXT3, contained more caftaric acid and coumaric acid but we did not find information about their potential impact on bone metabolism in the available data. Moreover, YL EXT3 proved the weakest antiosteoporotic activity in tests conducted as part of this study.

The article "A Comparison of the Antiosteoporotic Effects of Cornelian Cherry (Cornus mas L.) Extracts from Red and Yellow Fruits Containing Different Constituents of Polyphenols and Iridoids in Osteoblasts and Osteoclasts" was published in 2022. Journal: Oxid Med Cell Longev.

In previous studies, flavonols such as kaempferol and quercetin proved to have an antiosteoporotic effect. They decreased osteoclastogenesis, mainly through RANKL-related pathways, and promoted osteoblast differentiation [7, 52]. Proposed mechanisms responsible for the benefits of kaempferol in senile osteoporosis include also anti-inflammatory and antioxidative properties and regulation of osteoblasts' and osteoclasts' apoptosis [53]. Kaempferol and quercetin in the forms of 3-*O*-glucuronide, 3-*O*-galactoside, or *O*-glucoside were found in small amounts in RED EXT1, but their potential contribution to the antiosteoporotic effect is difficult to elucidate. YL EXT3 contained moderate amounts of quercetin 3-*O*-glucuronide but had the lowest antiosteoporotic potency. YL EXT2 did not contain flavonols. An accurate assessment of possible synergism between anthocyanin or iridoids and flavonols would require additional studies using different compositions of extracts and higher doses of flavonols.

Hydrolysable tannins were most abundant in RED EXT1, but substantial amounts were also found in YL EXT3; they were not present at all in YL EXT2. Previous studies have shown the antiosteoporotic potential of hydrolysable tannins. Corilagin inhibited osteoclastogenesis via downregulation of the NF-*κ*B and PI3K/AKT signaling pathways in murine bone marrow macrophage cells (BMMs) [54]. Other studies have proven that geraniin enhanced proliferation and osteoblastic differentiation of bone marrow-derived stem cells (BMSCs) in both normal and osteoporotic rats through the activation of Wnt/*β*-catenin signaling [55]; it also reduced bone turnover marker levels, increased osteoprotegerin (OPG), decreased RANKL, and increased the OPG/RANKL ratio in rats with ovariectomy-induced osteoporosis [9]. Hydrolysable tannins can also hydrolyze to phenolic acids, such as gallic acid and ellagic acid, and potentially exert an effect through these substances. Both RED EXT1 and YL EXT3 extracts were found to contain gemin, tellimagrandin, camptothin, and cornusiin isomers. It is worth emphasizing that cornusiin isomers were about 3 times more abundant in RED EXT1 than in YL EXT3. Although RED EXT1 proved to have strong antiosteoporotic effects, it is difficult to understand why YL EXT3 showed a lower efficacy than even YL EXT2, which did not contain any hydrolysable tannins at all. It is difficult to explain this finding, especially that we investigated mixtures of substances; contribution of hydrolysable tannins to antiosteoporotic effects may depend on its different structures and doses, and interactions with other extracts' constituents. It seems that among hydrolysable tannins detected in our study, the most promising substance is cornusiin, but further investigations with isolated compounds are needed.

The article "A Comparison of the Antiosteoporotic Effects of Cornelian Cherry (Cornus mas L.) Extracts from Red and Yellow Fruits Containing Different Constituents of Polyphenols and Iridoids in Osteoblasts and Osteoclasts" was published in 2022. Journal: Oxid Med Cell Longev.

Collectively, this study demonstrated that *Cornus mas L*. extracts enhanced osteoblastogenesis and reduced osteoclastogenesis. Comparison of the antiosteoporotic efficacy of the three extracts and analysis of the constituents in the polyphenols and iridoids, may help elucidate the molecular mechanisms responsible for the antiosteoporotic effects. Among the three extracts, the RED EXT1 extract uniquely comprised several anthocyanins and the highest variety of polyphenols and iridoids; the YL EXT2 extract uniquely contained gallic acid and the highest amount of an irodoid, loganic acid (Table 1). RED EXT1, and YL EXT2 showed similar efficacy to each other, and better efficacy than YL EXT3, in the augmentation of osteoblast differentiation (Figures 2–4). These results strongly suggest that the iridoids, such as loganic acid, present in the extracts, may be responsible for the increase in osteoblast differentiation via the upregulation of Alpl and Runx2 expressions at the transcription level. Meanwhile, RED EXT1 showed the best efficacy in inhibiting osteoclast differentiation (Figures 6–8), strongly suggesting that the anthocyanins present in the extracts may be responsible for the decrease in osteoclast differentiation via the downregulation of Nfatc1, Ctsk, and Acp5 expressions at the transcription level. A suggested molecular mechanism for *Cornus mas L.* extracts in the regulation of osteoblast and osteoclast differentiation is described in Figure 9.

## 4. Conclusions

The main conclusions of our study were that three extracts from red and yellow *Cornus mas* L. fruits containing different constituents of iridoids and polyphenols such as anthocyanins, hydrolysable tannins, phenolic acids, and flavonols had antiosteoporotic effects. All these extracts significantly enhanced osteoblast differentiation and significantly reduced osteoclast differentiation. The antiosteoporotic effects of the RED EXT1 extract, containing several anthocyanins and iridoids, exerted via reduction of osteoclast differentiation, were better than that of YL EXT2 and YL EXT3. These results suggest that the red *Cornus mas* L. extract could be a promising phytomedicine candidate for the prevention and treatment of osteoporosis.

The article "A Comparison of the Antiosteoporotic Effects of Cornelian Cherry (Cornus mas L.) Extracts from Red and Yellow Fruits Containing Different Constituents of Polyphenols and Iridoids in Osteoblasts and Osteoclasts" was published in 2022. Journal: Oxid Med Cell Longev.

## Figures and Tables

**Figure 1:** The effect of *Cornus mas* L. extracts on the cellular viability of primary osteoblasts in mice. Primary osteoblasts were incubated with ascorbic acid (50 *μ*g/mL), *β*-glycerophosphate (10 mM), and cotreated with RED EXT1 (a), YL EXT2 (b), and YL EXT3 (c) at three different concentrations (2, 5, and 10 *μ*g/mL) for 3 days. CM, *Cornus mas* L. extract. Cell viability was assessed using a water-soluble tetrazolium assay.

**Figure 2:** The effect of *Cornus mas* L. extracts on the alkaline phosphatase (ALP) activity in the primary osteoblasts of mice. The primary osteoblasts were incubated with ascorbic acid (50 *μ*g/mL), *β*-glycerophosphate (10 mM), and cotreated with RED EXT1 (a), YL EXT2 (b), and YL EXT3 (c) at three different concentrations (2, 5, and 10 *μ*g/mL) for three days. ALP activity was measured using p-nitrophenyl phosphate at an absorbance of 405 nm. CM, *Cornus mas* L. extract. ^∗^*p* < 0.05 vs. induction, ^#^*p* < 0.05 vs. CM2 (one-way analysis of variance (ANOVA) with Tukey's honest significant difference post hoc test).

**Figure 3:** The effects of *Cornus mas* L. extracts on alkaline phosphatase (ALP) staining in the primary osteoblasts of mice. The primary osteoblasts were incubated with ascorbic acid (50 *μ*g/mL) and *β*-glycerophosphate (10 mM) and cotreated with RED EXT1, YL EXT2, and YL EXT3 at three different concentrations (2, 5, and 10 *μ*g/mL) for 3 days. ALP-positive cells were visualized using a light microscope and indicated with arrows. CM, *Cornus mas* L. extract.

**Figure 4:** The effects of the *Cornus mas* L. extracts on the expression changes of osteoblast-specific genes in the primary osteoblasts of mice. The primary osteoblasts were incubated with ascorbic acid (50 *μ*g/mL) and *β*-glycerophosphate (10 mM) with or without 10 *μ*g/mL of *Cornus mas* L. extracts for 3 days. Osteoblast-specific genes including Alpl and Runx2 were measured by qRT-PCR using gene-specific primers. CM, *Cornus mas* L. extract treatment. ^∗^*p* < 0.05 vs. induction (Student's *t*-test).

**Figure 5:** The effect of *Cornus mas* L. extracts on the cellular viability of primary osteoclasts in mice. The primary monocytes were incubated with macrophage colony-stimulating factor (M-CSF) (50 ng/mL) and receptor activator of nuclear factor-kappa B ligand (RANKL) (50 ng/mL) and cotreated with RED EXT1 (a), YL EXT2 (b), and YL EXT3 (c) at three different concentrations (2, 5, and 10 *μ*g/mL) for 5 days. Cell viability was assessed using a WST assay. CM, *Cornus mas* L. extract.

The article "A Comparison of the Antiosteoporotic Effects of Cornelian Cherry (Cornus mas L.) Extracts from Red and Yellow Fruits Containing Different Constituents of Polyphenols and Iridoids in Osteoblasts and Osteoclasts" was published in 2022. Journal: Oxid Med Cell Longev.

**Figure 6:** The effect of *Cornus mas* L. extracts on tartrate-resistant acid phosphatase (TRAP) activity in the primary osteoclasts of mice. The primary monocytes were incubated with M-CSF (50 ng/mL) and RANKL (50 ng/mL) and cotreated with RED EXT1 (a), YL EXT2 (b), and YL EXT3 (c) at three different concentrations (2, 5, and 10 *μ*g/mL) for 5 days. TRAP activity was measured using acid-phosphatase at an absorbance of 405 nm. CM, *Cornus mas* L. extract. ^∗^*p* < 0.05 vs. induction, ^#^*p* < 0.05 vs. CM2, ^$^*p* < 0.05 vs. CM5 (one-way ANOVA with Tukey's honest significant difference post hoc test).

**Figure 7:** The effects of *Cornus mas* L. extracts on the tartrate-resistant acid phosphatase (TRAP) staining of primary osteoclasts in mice. The primary monocytes were incubated with ascorbic acid (50 *μ*g/mL) and *β*-glycerophosphate (10 mM) and cotreated with RED EXT1, YL EXT2, and YL EXT3 at three different concentrations (2, 5, and 10 *μ*g/mL) for 5 days. TRAP-positive cells were visualized using a light microscope and indicated with arrows. CM, *Cornus mas* L. extract.

**Figure 8:** The effects of *Cornus mas* L. extracts on the expression changes of osteoclast-specific genes in the primary osteoclasts of mice. The primary monocytes were incubated with M-CSF (50 ng/mL) and RANKL (50 ng/mL) with or without 10 *μ*g/mL of *Cornus mas* L. extracts for 5 days. Osteoclast-specific genes including Nfatc1, Ctsk, and Acp5 were measured with qRT-PCR using gene-specific primers. CM; *Cornus mas* L. extract. ^∗^*p* < 0.05 vs. induction (Student's *t*-test).

**Figure 9:** A suggested molecular mechanism for *Cornus mas* L. extracts in the regulation of osteoblast and osteoclast differentiation. Abbreviations: M-CSF, macrophage colony-stimulating factor; OPG, osteoprotegerin; RANKL, receptor activator of nuclear factor-kappa B ligand.

**Table 1:** Identification and content (mg/100 g dw) of main compounds of extracts from red (RED EXT1) and yellow (YL EXT2 and YL EXT3) cornelian cherry fruits by using LC-MS and HPLC.

Compound	UV *λ*_max_	MS^1^ [M − H]^–^/[M − H]^+^	MS^2^ Other ions	RED EXT1	YL EXT2	YL EXT3
	(nm)	(*m/z*)	(*m/z*)	Mg/100 g DW		
*IRIDOIDS*						
Loganic acid	245	375	213	12913.51 ± 159.09	22052.09 ± 206.67	17986.41 ± 190.37
Sweroside	245	403 [M − H + 46]^−^	195	533.64 ± 14.71	0.00	1135.86 ± 15.95
Loganin	245	435 [M − H + 46]^−^	227	1285.98 ± 35.44	0.00	2205.69 ± 30.97
Cornuside	245/273	541	169	2140.49 ± 17.96	0.00	6364.23 ± 50.54
Total iridoids				**16873.62**	**22052.09**	**27692.19**
*ANTHOCYANINS*						
Delphinidin 3-*O*-galactoside	524	463+	303+	663.84 ± 7.42	0.00	0.00
Cyanidin 3-*O*-galactoside	515	449+	287+	203.43 ± 8.49	0.00	0.00
Cyanidin 3-*O*-robinobioside	516	595+	287+	301.25 ± 3.26	0.00	0.00
Pelargonidin 3-*O*-galactoside	501	433+	271+	1509.59 ± 23.75	0.00	0.00
Pelargonidin 3-*O*-robinobioside	501	579+	271+	268.22 ± 7.44	0.00	0.00
Cyanidin	523	287+		231.34 ± 6.01	0.00	0.00
Pelargonidin	509	271+		300.75 ± 5.47	0.00	0.00
Total anthocyanins				**3478.42**	**0.00**	**0.00**
*PHENOLIC ACIDS*						
Gallic acid	272	169		0.00	263.59 ± 9.94	0.00
*Trans*-caftaric acid	326	311	179/149	101.03 ± 5.76	252.58 ± 4.47	43.63 ± 3.42
Caftaric acid isomer	326	311	179/149	562.26 ± 9.56	360.82 ± 13.68	1102.77 ± 27, 14
Coutaric acid isomer	312	295	163/149	333.07 ± 8.82	36.08 ± 2.19	1475.38 ± 36.47
*p*-Coumaric acid	310	163		33.58 ± 1.70	0.00	565.88 ± 12.78
Ellagic acid	254	301		146.24 ± 1.06	0.00	338,53 ± 7.92
Total phenolic acids				**1176.18**	**913.07**	**3526.19**
*FLAVONOLS*						
Quercetin 3-*O*-glucuronide	354	477	301	306.24 ± 10.42	0.00	816.52 ± 13.52
Quercetin 3-*O*-glucoside	353	463	301	23.69 ± 2.07	0.00	0.00
Kaempferol 3-*O*-galactoside	348	447	285	235.32 ± 9.97	0.00	0.00
Kaempferol 3-*O*-glucuronide	351	461	285	27.93 ± 2.76	0.00	0.00
Total flavonols				**593.18**	**0.00**	**816.52**
*HYDROLYSABLE TANNINS*						
Total gemin D isomers	265	633	301/275/249/169	903.33	0.00	1024.41
Tellimagrandin I	267	785	633/301/275/249/169	276.11	0.00	437.58
Tellimagrandin II	271	937	785/633/301/275/249/169	595.47	0.00	0.00
Total camptothin A isomers	264	708^−2^, 1417	1247/783/633/301	2294.22	0.00	2699.29
Total cornusiin A isomers	273	784^−2^, 1569	935/633/313/301	8503.24	0.00	3385.07
Total cornusiin C isomers	268	1176^−2^, 2353	786/633/451/301	4249.05	0.00	1551.42
Total hydrolysable tannins				**16821.42**	**0.00**	**9097.77**

Abbreviations: (dw): dry weight; (HPLC): high-performance liquid chromatography; (LC-MS): liquid chromatography-mass spectrometry; (*m/z*): mass-to-charge ratio.

The article "A Comparison of the Antiosteoporotic Effects of Cornelian Cherry (Cornus mas L.) Extracts from Red and Yellow Fruits Containing Different Constituents of Polyphenols and Iridoids in Osteoblasts and Osteoclasts" was published in 2022. Journal: Oxid Med Cell Longev.

## Data Availability

All the data generated or analyzed during this study are included in this article. Further inquiries can be directed to the corresponding authors.

## Abbreviations

Acp5: Tartrate-resistant acid phosphatase 5
ALP: Alkaline phosphatase
Alpl: Alkaline phosphatase, biomineralization associated
Bglap: Bone gamma-carboxyglutamic acid-producing protein
CM: *Cornus mas*
CtsK: Cathepsin K
Dw: Dry weight
ESI: Electrospray ionization
ERK 1/2: Extracellular signal-regulated protein kinase 1/2
GSK-3*β*: Glycogen synthase kinase 3 beta
HPLC–PDA: High-performance liquid chromatography–photodiode array detection
LC-MS: Liquid chromatography mass spectrometry
M-CSF: Macrophage colony-stimulating factor
*M/z*: Mass-to-charge ratio
Nfatc1: Nuclear factor of activated T cells 1
NF-*κ*B: Nuclear factor kappa-light-chain-enhancer of activated B cells
OPG: Osteoprotegerin
PI3K/AKT: Phosphatidylinositol 3-kinase/protein kinase B
PPARs: Peroxisome proliferator-activated receptors
RANKL: Receptor activator of nuclear factor-kappa B ligand
qRT-PCR: Quantitative reverse transcriptase-polymerase chain reaction
Q-TOF: Quadruple time of flight
Runx2: Runt-related transcription factor 2
TRAP: Tartrate-resistant acid phosphatase
UPLC: Ultra-performance liquid chromatography.
